# Calycosin Inhibits the Malignant Behaviors of Lung Adenocarcinoma Cells by Regulating the circ_0001946/miR-21/GPD1L/HIF-1*α* Signaling Axis

This article has been retracted.

**DOI:** 10.1155/2022/3969389

**Published:** 2022-08-13

**Authors:** Lixia Zhou, Wenxian Chen, Hang Yang, Jiaqin Liu, Hui Meng

**Affiliations:** ^1^Department of Oncology, The Fifth Affiliated (Zhuhai) Hospital of Zunyi Medical University, Zhuhai, Guangdong 519100, China; ^2^Department of Thoracic Surgery, The Fifth Affiliated (Zhuhai) Hospital of Zunyi Medical University, Zhuhai, Guangdong 519100, China

## Abstract

**Objective:**

To clarify the potential function and molecular mechanism of calycosin in lung adenocarcinoma (LUAD) cells.

**Methods:**

LUAD cells (A549 and H1299) were treated with calycosin at different concentrations (25 nM, 50 nM, and 100 nM) for 24 h. The colony formation, invasion, and migration of the cells were assessed by colony formation, transwell, and scratch assays, respectively. Quantitative reverse transcription-polymerase chain reaction (qRT-PCR) was performed to determine the mRNA expression level of circ_0001946, miR-21, glycerol-3-phosphate dehydrogenase 1 like (GPD1L), and hypoxia-inducible factor-1*α* (HIF-1*α*) in clinical tissue samples and LUAD cells. RNA pull-down assay and dual-luciferase reporter assay were performed to verify the relationship among circ_0001946, miR-21, GPD1L, and HIF-1*α*. Western blot was performed to detect the protein expression of epithelial-mesenchymal transition (EMT) process-related genes (E-cadherin, N-cadherin, and snail) and GPD1L as well as HIF-1*α*.

**Results:**

Calycosin inhibited colony formation, invasion, migration, and EMT progression in A549 and H1299 cells. Besides, calycosin was able to regulate the expression of circ_0001946, miR-21, GPD1L, and HIF-1*α* in LUAD cells. According to the findings of QRT-PCR, the expression level of circ_0001946 and GPD1L in LUAD tissues was significantly lower than that in adjacent noncancerous normal tissues, and the expression of miR-21 and HIF-1*α* was also significantly increased in clinical tissue samples. In addition, there was a targeted regulatory relationship among the above four expressions. Knockdown of circ_0001946 expression in A549 cells treated with calycosin enhanced the malignant behavior of A549 cells and inhibited the anticancer effect of calycosin. However, the knockdown of miR-21 promoted the anticancer effect of calycosin and inhibited the malignant behavior of A549.

**Conclusion:**

Calycosin can inhibit colony formation, invasion, migration, and EMT process of LUAD cells via regulating the circ_0001946/miR-21/GPD1L/HIF-1*α* signaling axis and could be a promising therapeutic drug for LUAD.

## 1. Introduction

As one of the cancers with the highest malignant degree, lung cancer is accompanied by a 4%-17% 5-year survival rate, making it the most common cause of cancer-related death worldwide [1]. Non-small-cell lung cancer (NSCLC) accounts for nearly 80% of lung cancers, including about 50% of lung adenocarcinoma (LUAD). The prevalence of LUAD is increasing annually and is about to become the main subtype of NSCLC [2]. Despite improvements in early diagnosis, patients with LUAD still have a low 5-year overall survival rate and unsatisfactory recurrence rate [3, 4]. Currently, the clinical treatment protocols for LUAD mainly include drugs and radiotherapy; however, they are often prone to tolerance in patients [5]. It was reported that when treated with EGFR tyrosine kinase inhibitors (TKIs), gefitinib or erlotinib and osimertinib, most LUAD patients with EGFR mutations acquired drug resistance mutations [6]. Hence, it is essential to explore new therapeutic agents and elucidate their molecular mechanisms to develop new therapeutic strategies to treat LUAD.

Circular RNA (circRNA), an endogenous noncoding RNA with a covalently closed-loop structure but without a 5′ cap and 3′ polyadenylate tail, is resistant to exonucleases [7]. A large number of previous studies have confirmed the presence of circRNAs in a variety of diseases and cancers [8]. Some reports revealed the involvement and different roles of many circRNAs in the development of LUAD. For example, high circ_0023404 expression was shown to be associated with poor prognosis in lung cancer patients [9]. In addition, circ-RAD23B can promote cell growth and metastasis in NSCLC [10]. Relevant articles have indicated that circ_0001946 expression is downregulated in various cancers, such as the case of bladder cancer and glioblastoma [11]. Huang et al. [12] discovered that circRNA has_circ_0001946 inhibited lung cancer progression and mediated NSCLC cisplatin sensitivity through nucleotide excision repair. Notably, Yao et al. [13] claimed that circ_0001946 was also involved in LUAD development and was a potential biomarker for treating LUAD. It can be seen that circRNA is of vital significance in tumor progression, and circ_0001946 may be a potential target for the treatment of lung cancer. Further exploration is required for circ0001946 due to its complex function.

Great progress has been achieved in using extracts of traditional Chinese medicine (TCM) in treating cancer, which has emerged as a potential cancer therapy. Calycosin, a fat-soluble component in radix astragali (the dried roots of *Astragalus membranaceus*), is a commonly seen organic compound in nature, with antioxidant and anti-inflammatory properties [14]. Recently, calycosin has attracted much attention due to the discovery of its anticancer effects. Wang et al. [15] found that calycosin inhibited the invasion and metastasis of colorectal cancer cells by regulating the epithelial-mesenchymal transition (EMT) of cells. Zhang et al. [16] proved that calycosin could inhibit pancreatic cancer cell growth by inducing cell cycle arrest and apoptosis and induce the metastatic progression of pancreatic cancer by regulating the tumor microenvironment. Through the above findings, it can be speculated that calycosin is a potential anticancer drug. However, there are few studies on calycosin's role in treating LUAD. At present, Cheng et al. [17] discovered that calycosin was able to inhibit the proliferation and metastasis of human LUAD cells (A549). However, the mechanism of action of calycosin in inhibiting cancer remains to be uncovered, urging in-depth study.

Given the above limitations in literature, in this study, we attempted to investigate the effect and underlying mechanisms of calycosin on the progression of LUAD cells, including the effect on the expression and function of circ_0001946, with the aim of suggesting the potential significance of calycosin as a promising agent for the treatment of LUAD.

## 2. Materials and Methods

### 2.1. Clinical Sample Collection

Tumor tissues (LUAD) and histologically normal tissue (normal) were collected from 20 LUAD patients who underwent surgery at The Fifth Affiliated (Zhuhai) Hospital of Zunyi Medical University between June 2018 and December 2020. This study was approved by the Research Ethics Committee of The Fifth Affiliated (Zhuhai) Hospital of Zunyi Medical University (approval number: 2022ZH060), and all experiments were conducted following approved guidelines. The patients gave informed consent for tissue specimen collection and voluntarily signed the informed consent form. Samples were frozen in liquid nitrogen immediately and stored at -80°C prior to use.

### 2.2. Cell Culture and Treatment

Human normal lung epithelial cells BEAS-2B and human LUAD cells A549 and H1299 were purchased from the National Collection of Authenticated Cell Cultures. BEAS-2B, A549, and H1299 cells were cultured in DMEM (Hyclone, USA) containing 10% fetal bovine serum (FBS, Gibco, USA), 100 mg/mL penicillin, and 100 mg/mL streptomycin. The medium was placed in an incubator with 5% CO_2_ at 37°C.

A549 and H1299 cells were treated with 25 nM, 50 nM, and 100 nM calycosin [15] for 24 h when the confluence reached 65%-80%. Then, subsequent functional assays were conducted. The circ_0001946 interfering fragment (si-circ_0001946) and its control (si-NC), miR-21 mimics and its control (miR-21 NC), and miR-21 inhibitor and its control inhibitor were designed and synthesized by GenePharma (Shanghai, China). Cells were seeded and cultured in 6-well plates until their confluence reached 65%-80%. Subsequently, the above fragments or vectors were transfected into A549 and H1299 cells using Lipofectamine 2000 (Invitrogen, USA). After 48 h culture, the cells were collected. In addition, to verify the action mechanism of calycosin, A549 cells were first treated with 100 nM calycosin for 24 h and then transfected with miR-21 inhibitor and si-circ0001946.

### 2.3. Cell Cloning Assay

Cells with different treatments in the logarithmic growth phase were seeded in a 6-well cell culture plate at 500 cells/well; then, an incubator with 5% CO_2_ was applied for cell culture at 37°C for approximately 14 days. Next, the cells were gently rinsed with PBS solution, fixed with 4% paraformaldehyde (Beyotime, China) for 30 min, and stained with crystal violet staining solution (Beyotime, China) for 10-30 min. Finally, the excess staining solution was washed off with PBS solution, and the number of colony formations was counted.

### 2.4. Transwell

Matrigel was dissolved at 4°C and diluted according to a certain proportion. Then, the diluted Matrigel was added to the bottom of the transwell chamber and solidified in an incubator at 37°C. The cells in the logarithmic growth phase were digested and collected. After resuspension with a serum-free DMEM, the concentration of cell suspension was adjusted to 8 × 10^5^ cells/mL. Subsequently, 100 *μ*L of cell suspension was added to the transwell insert plated with Matrigel, and 600 *μ*L of DMEM with 20% FBS was added to the lower chamber. Then, an incubator was used for incubation at 37°C for 20-24 h. After that, the insert was removed, and 4% paraformaldehyde was added for 30 min fixation. A cotton swab was used to wipe off residual cells in the insert; then, crystal violet staining solution was added for staining for 10-30 min. After the completion of staining, PBS solution was employed to wash off the excess staining solution. Under the microscope, random 5 fields were selected for picture collection and cell counting.

### 2.5. Scratch Assay

The cells were seeded into 6-well plates at the density of 1 × 10^6^ cells/well and incubated overnight to reach confluence. The scratch was created with a pipette tip, and the floating cells were cleared with PBS. Then, the scratch was imaged under a microscope after 0 h and 12 h of culture in an incubator at 37°C. The scratch area was determined using ImageJ software, and the migration rate was calculated according to the migration area calculation formula: migration rate = (A0 − An)/A0, with A0 representing the initial scratch area and An representing the scratch area after 12 h.

### 2.6. Western Blot

The total protein was extracted from the cells with RIPA Lysing Solution (Beyotime, China) and then quantified by a BCA kit (Beyotime, China). Subsequently, 30 *μ*L of total protein was separated by sodium dodecyl sulfate-polyacrylamide gel electrophoresis (SDS-PAGE) and transferred to a polyvinylidene fluoride (PVDF) membrane. Next, the membrane was blocked with 5% skimmed milk for 1-3 h at ambient temperature and then incubated with primary antibodies (anti-E-cadherin, anti-N-cadherin, anti-Snail, anti-HIF-1*α*, anti- GPD1L, and anti-*β*-actin, CST, USA) overnight at 4°C. Later, the membrane was washed three times with PBST and incubated with horseradish peroxidase-conjugated secondary antibodies (CST, USA) for 1 h at ambient temperature. Immunoreactive bands were developed using enhanced chemiluminescence reagents (Thermo, USA) and imaged by a ChemiDoc XRS Plus luminescent image analyzer (Bio-Rad). The grayscale was analyzed using Image-Pro Plus 6.0 software, and the relative expression level of the proteins was calculated with *β*-actin as an internal control due to its high stability as a housekeeping gene.

### 2.7. qRT-PCR

TRizol method (Solarbio, China) was employed to extract total cellular and tissue RNA, followed by the detection of the concentration and purity of RNA with NanoDrop. Then, RNA was utilized to prepare cDNA according to the instructions of the random primer reverse transcription kit (Thermo, USA). The expression level of circ_0001946, miR-21, GPD1L, and HIF-1*α* in the cells was measured per the instructions of the SYBR Green kit (TaKaRa, Japan). U6 and GADPH served as internal controls, and six replicates were set up in the experiment. The experimental data obtained by qRT-PCR were used to calculate the relative expression of the target gene with the 2 ˉ^*ΔΔ*Ct^ method. Primer sequences are displayed in Table 1.

### 2.8. RNA Pull-Down Assay

A549 and H1299 cells were harvested and lysed by sonication. Biotinylated miR-21-bio and its control (miR-21-bio NC) were constructed, and biotinylated RNA was incubated with cell lysate at 4°C overnight. Agarose beads were then added for another 1 h incubation, and the expression of circ_0001946 in the precipitated complex was detected with qRT-PCR.

### 2.9. Dual-Luciferase Reporter

The sequence containing circ_0001946 wild-type (circ_0001946WT) or circ_0001946 mutant (circ_0001946-MUT) and the sequence containing GPD1L wild-type (GPD1LWT) or GPD1L mutant were constructed into the dual-luciferase reporter plasmid (GP-miRGLO). miR-21 mimics or miR-21 NC were cotransfected into HEK-293T cells with a luciferase reporter plasmid. After 48 h, the luciferase activity was measured using the Dual-Luciferase Reporter System Kit (E1910, Promega, USA).

### 2.10. Data Analysis

The results are expressed as mean ± standard deviation (SD). The SPSS v26.0 and Graphpad Prism v9.0 software were used for statistical analysis. One-way analysis of variance was used for comparison between multiple groups and an independent sample *T*-test for comparison between two groups. Pearson correlation was applied to analyze the expression correlation, and *p* < 0.05 was used to determine statistical significance.

## 3. Results

### 3.1. Calycosin Inhibits Colony Formation, Invasion, Migration, and Epithelial-Mesenchymal Transition in Lung Adenocarcinoma Cells

Calycosin is a natural compound with antioxidant and estrogenic activity, which has anticancer potential (Figure 1(a)). To explore the role of calycosin in LUAD, we treated LUAD cells (A549 and H1299) with different concentrations of calycosin (25 nM, 50 nM, and 100 nM). The colony formation, invasion, and migration ability of cells in each group were tested by cell colony formation, transwell, and scratch assays, respectively. The results revealed that the abilities of colony formation (Figures 1(b)–1(c)), invasion (Figures 1(d) and 1(e)), and migration (Figures 1(f) and 1(g)) of A549 and H1299 cells in the CA 25 nM group, CA 50 nM group, and CA 100 nM group were all significantly reduced in a concentration-dependent manner compared with the control group (*p* < 0.01). Additionally, to understand the effects of calycosin on the EMT process of LUAD, we examined the expression level of EMT-related proteins in cells of each group using western blot. The results showed that calycosin could significantly increase the protein expression level of E-cadherin and decrease the level of N-cadherin and Snail in A549 and H1299 cells in a concentration-dependent manner (Figures 1(h)–1(j)). In summary, calycosin could significantly inhibit colony formation, invasion, migration, and EMT progression of LUAD cells.

### 3.2. Calycosin Upregulates circ_0001946 Level in Lung Adenocarcinoma Cells

Aside from the above finding, we also discovered that calycosin could significantly increase the expression level of circ_0001946 in A549 and H1299 cells in LUAD in a concentration-dependent manner (*p* < 0.01, Figures 2(a) and 2(b)). However, it remained unclear whether calycosin inhibited LUAD cell colony formation, invasion, migration, and EMT process through circ_0001946. To figure this out, the expression of circ_0001946 in LUAD was examined by qRT-PCR. The results showed that the expression level of circ_0001946 in LUAD tissues was much lower than that in normal tissues (*p* < 0.01, Figure 2(c)); and similar results were also observed at the cellular level; that is, the expression level of circ_0001946 in A549 and H1299 cells in LUAD was significantly decreased compared with that in normal lung epithelial cells BEAS-2B (*p* < 0.01, Figure 2(d)). These results suggested that calycosin could inhibit the malignant behaviors of LUAD cells by upregulating circ_0001946.

### 3.3. circ0001946 Can Serve as a Sponge for miR-21

circRNAs can regulate signal transmission through molecular sponge microRNAs. However, it remained unknown whether upregulated circ_0001946 after calycosin treatment could play its role by sponging microRNAs. To verify this, miR-21 was predicted as a downstream target of circ_0001946 by bioinformatics analysis (Starbase.2). After calycosin treatment, the expression of miR-21 in A549 and H1299 cells was examined. The results showed that calycosin treatment was able to significantly downregulate the expression of miR-21 (Figures 3(a) and 3(b)), suggesting that calycosin could upregulate circ_0001946 by sponging miR-21. The expression of miR-21 in clinical samples was further evaluated, and the results indicated that miR-21 expression level in LUAD tissues was significantly elevated compared with adjacent normal tissues (*p* < 0.01, Figure 3(c)). Additionally, miR-21 expression was negatively correlated with circ_0001946 expression in LUAD tissues (Figure 3(d)). Therefore, we speculated that there was a targeting relationship between circ_0001946 and miR-21. Subsequently, the binding sites of miR-21 and circ0001946 were predicted, and the prediction outcomes are shown in Figure 3(e). Next, a luciferase reporter assay was performed in 293T cells to assess the relationship between miR-21 and circ0001946. According to the results, compared with the MUT group, cells in the WT group treated with miR-21 mimics presented lower luciferase activity (Figure 3(f)). RNA pull-down assay presented that circ_0001946 could bind to miR-21 (Figures 3(g) and 3(g)). After knockdown of circ_0008035 expression in A549 and H1299 cells by si-circ0001946, miR-21 expression in the cells was significantly increased compared with the siNC group (*p* < 0.01, Figures 3(i)–3(l)). In summary, our results showed that circ0001946 could be used as a sponge for miR-21.

### 3.4. miR-21 Can Target GPD1L

As a microRNA, miR-21 can target and bind mRNA to regulate the expression of genes and then exert biological functions. It could be observed in this study that calycosin was able to significantly increase GPD1L expression levels in A549 and H1299 cells (*p* < 0.01, Figures 4(a) and 4(b)). Then, the binding sites of miR-21 and GPD1L were predicted, and the specific results are shown in Figure 4(c). The targeting relationship between miR-21 and GPD1L was verified by a dual-luciferase reporter assay. Compared with the GPD1L-MUT group, we observed a much lower luciferase activity of cells in the GPD1L-WT group after the treatment of miR-21 mimics (Figure 4(d)). Subsequently, a negative correlation between miR-21 expression and GPD1L expression was discovered in LUAD clinical samples (Figure 4(e)). In addition, knockdown of miR-21 in A549 or H1299 cells was able to significantly upregulate the mRNA and protein expression level of GPD1L (Figures 4(f)–4(k)). The above findings suggested that GPD1L was a potential target gene of miR-21.

### 3.5. miR-21 Regulates the Level of HIF-1*α* through GPD1L

Interestingly, the level of bHLH-PAS family transcription factor HIF-1*α* in A549 and H1299 cells after calycosin treatment was significantly reduced compared with that in the control group in this study (*p* < 0.01, Figures 5(a) and 5(b)). This result suggested that calycosin could regulate the level of HIF-1*α* in LUAD cells. In addition, after the knockdown of miR-21 and GPD1L (miR-21 inhibitor+si-GPD1L), the miR-21 inhibitor group exhibited significantly decreased HIF-1*α* expression levels in both A549 and H1299 cells, while the mRNA and protein expression levels of HIF-1*α* in cells of the miR-21 inhibitor+si-GPD1L group were significantly downregulated compared with those in the miR-21 inhibitor group (Figures 5(c)–5(f)). Moreover, a negative correlation was observed between the expression of GPD1L and HIF-1*α* in LUAD clinical tissues (Figure 5(g)). Taken together, miR-21 regulated HIF-1*α* expression through GPD1L.

### 3.6. Calycosin Regulates Colony Formation, Invasion, Migration, and EMT of Lung Adenocarcinoma Cells through the circ0001946/miR-21/GPD1L/HIF-1*α* Signaling Axis

To determine whether calycosin inhibited the malignant behavior of LUAD cells through the circ_0001946/miR-21/GPD1L/HIF-1*α* signaling axis, the cells treated by calycosin were transfected with si-circ0001946 or miR-21 inhibitor. Then, the abilities of colony formation, invasion, migration, and EMT process of A549 cells were assessed by colony formation assay, transwell, scratch assay, and western blot. The results are shown in Figure 6. We observed that compared with the CA group, the CA+si-circ_0001946 group presented a significant increase in colony formation, invasion, and migration abilities of A549 cells (*p* < 0.01), and at the same time, the EMT process of cells was also promoted (downregulation of E-cadherin, upregulation of N-cadherin and snail). When treatment with calycosin and transfection with miR-21 inhibitor (CA+inhibitor group) were performed simultaneously, the above phenotypes of A549 cells were reversed, showing markedly reduced abilities of colony formation, invasion, migration, and EMT process of A549 cells (*p* < 0.01, Figures 6(a)–6(f)). In addition, the GPD1L expression level in A549 cells in the CA+si-circ0001946 group was much lower than that in the CA group, while the level of HIF-1*α* was notably increased. The expression level of GPD1L in cells of the CA+inhibitor group was significantly increased compared with that of the CA group, while the level of HIF-1*α* was significantly decreased (Figures 6(i)–6(l)). In summary, the circ0001946/miR-21/GPD1L/HIF-1*α* signaling axis was a key mediator of the anticancer function exerted by calycosin.

## 4. Discussion

In previous studies, Chinese herbal extracts have attracted researchers' interests due to their satisfactory anticancer properties, such as inhibiting cancer cell growth, proliferation, and differentiation [18]. Calycosin is a natural isoflavone isolated from *Astragalus membranaceus*, with anti-inflammatory, antioxidant, and antitumor properties. Li et al. [19] reported that calycosin inhibited migration and invasion of human breast cancer cells by downregulating the expression of Foxp3. In addition, calycosin was shown to inhibit osteosarcoma cell migration and invasion [19]. In this study, it was demonstrated that calycosin could inhibit the proliferation, migration, invasion, and EMT progression of LUAD cells (A549, H1299) in a dose-dependent manner. These were generally consistent with the findings of Zhang et al. in breast cancer cells [20], indicating that calycosin could exert an inhibitory role in the progression of LUAD.

Recent studies have shown that cancer development is significantly correlated with the expression of noncoding RNAs [21]. Specifically, abnormal circRNA levels may affect the expression of specific genes and cause tumorigenesis or tumor progression [21]. Among circRNAs, circ_0001946 has been determined to involve various cancers, including LUAD [12]. Our study presented significantly downregulated circ0001946 expression in LUAD tumor tissues collected clinically, while calycosin could significantly upregulate circ_0001946 expression. Yao et al. [13] reported that circ_0001946 was significantly upregulated in LUAD tumor tissues, but Zhang et al. [22] found that the median expression level of circ_0001946 in NSCLC tissues was more than 3 times higher than that in tumor tissues. Besides, the expression of circ_0001946 in tumor tissues was also significantly lower than in tumor tissues in esophageal adenocarcinoma (ESCC) [23]. All in all, it is inconclusive whether circ_0001946 plays an anticancer or inhibitory role in malignant tumors since its expression may be affected by various factors.

It is reported that circRNAs can regulate biological processes through various action mechanisms, including “miRNA sponges,” transcriptional regulation, protein binding, and translation [24]. Thereinto, miRNAs, small noncoding RNAs containing about 22 nucleotides, can regulate the expression of downstream target genes at the posttranscriptional level. According to recent studies, miRNAs are implicated in several physiological processes as well as tumorigenesis and metastasis of cancer [25, 26]. Moreover, it was revealed that miR-21 is overexpressed in most cancers and plays a key role in cancer progression. For instance, Wang et al. [27] showed that miR-21 promoted LUAD cell proliferation, migration, and invasion by targeting WWC2. Du et al. [28] discovered that miR-21-5p promoted LUAD progression by regulating PIK3R1 expression. In this study, the significantly elevated expression level of miR-21 was observed in LUAD tumor samples, while calycosin could significantly downregulate the expression of miR-21. Aside from this, circ_0001946 showed a negative correlation with the expression of miR-21. Moreover, circ_0001946 could be used as a sponge of miR-21 via dual luciferase and RNA pull-down assays.

Reprogrammed energy metabolism is one of the hallmarks of cancer. Under aerobic glycolysis, cancer cells show glycolysis rather than oxidative phosphorylation, even in the presence of oxygen. Cancer cells can stop glycolysis to promote survival, growth, metastasis, stemness, drug resistance, long-term maintenance, and immune evasion of cancer cells [29]. Preceding studies have confirmed the presence of transcriptional regulators of aerobic glycolysis in cancer, for example, HIF-1*α*, c-MYC, and p53 [30]. GPD1L is a mediator involved in regulating aerobic glycolysis and can act as a tumor suppressor in cancer. It was shown that GPD1L inhibited prolyl hydroxylase activity and could hydroxylate proline in HIF-1*α* to promote its proteasomal degradation, thus exerting anticancer activity [31]. This study also revealed that miRNAs regulated GPD1L. Du et al. found that upregulated miR-210-3p in triple-negative breast cancer (TNBC) could target and inhibit the expression of GPD1L, then promote aerobic glycolysis in cells [32]. In this study, GPD1L expression was regulated by calycosin and miR-21, and a targeting relationship could be observed between miR-21 and GPD1L. After further investigation, miR-21 was found to be able to regulate HIF-1*α* level through GPD1L. Subsequently, *in vitro* experiments with knockdown of circ_0001946/miR-21 also confirmed that calycosin could regulate the proliferation, invasion, migration, and EMT of LUAD cells through the circ_0001946/miR-21/GPD1L/HIF-1*α* signaling axis. Nevertheless, the exact mechanism of calycosin affecting the expression of circ_0001946 remains unclear up till now. In addition, we only researched the function and mechanism of calycosin in cells; thus, *in vivo* experiments and more studies are required to validate our findings and provide a more comprehensive theoretical basis for the clinical application of calycosin.

## 5. Conclusion

Calycosin inhibited colony formation, invasion, migration, and EMT progression of LUAD cells through the circ_0001946/miR-21/GPD1L/HIF-1*α* signaling axis in a concentration-dependent manner and demonstrated the potential to be an effective therapeutic agent for the treatment of LUAD.

## Figures and Tables

**Figure 1:** Calycosin inhibits the abilities of colony formation, invasion, migration, and EMT progression in lung adenocarcinoma cells. (a) Chemical formula of calycosin. (b–g) The effect of different concentrations of calycosin on the colony formation (b, c), invasion (d, e), and migration (f, g) abilities of A549 and H1299 cells was assessed by colony formation assay (b, c), transwell (d, e), and scratch assay (f, g), respectively. (h–j) The effect of calycosin on the expression of EMT-related proteins (E-cadherin, N-cadherin, and Snail) detected by western blot, ^∗∗^*p* < 0.01*vs.* control.

**Figure 2:** Calycosin upregulates circ_0001946 levels in lung adenocarcinoma cells. (a, b) The effects of different concentrations of calycosin on the expression of circ_0001946 in A549 (a) and H1299 (b) cells detected by qRT-PCR. (c) The expression of circ0001946 in clinical LUAD tissues and normal tissues determined by qRT-PCR. (d) The expression of circ0001946 in human normal lung epithelial cells BEAS-2B and human LUAD cells A549 and H1299 detected by qRT-PCR, ^∗∗^*p* < 0.01*vs.* control.

**Figure 3:** circ_0001946 can serve as a sponge for miR-21. (a, b) The effect of different concentrations of calycosin on the expression of miR-21 in A549 (a) and H1299 (b) detected by qRT-PCR. (c) The expression of miR-21 in clinical tissue samples (LUAD and normal tissues) detected by qRT-PCR. (d) The correlation between the expression of circ_0001946 and miR-21 in clinical LUAD tissues analyzed by Pearson analysis. (e) Prediction of the targeting sequence of miR-21 and GPD1L. (f) The targeting relationship between circ_0001946 and miR-21 validated by dual-luciferase assay. (g, h) The binding of circ_0001946 to miR-21 in A549 (g) and H1299 (h) cells assessed by RNA pull-down assay. (i, j) The knockdown efficiency of si-circ0001946 on circ_0001946 in A549 (i) and H1299 (j) cells. (k, l) miR-21 expression in A549 (k) and H1299 (l) after knockdown of circ_0001946 detected by qRT-PCR, ^∗∗^*p* < 0.01*vs.* control.

**Figure 4:** miR-21 can target GPD1L. (a, b) The effect of different concentrations of calycosin on GPD1L expression in A549 and H1299 cells observed via qRT-PCR, ^∗∗^*p* < 0.01*vs.* control. (c) Targeting sequence prediction of miR-21 and GPD1L. (d) The target relationship between miR-21 and GPD1L verified by dual-luciferase assay, ^∗∗^*p* < 0.01*vs.* GPD1LMUT. (e) The correlation between miR-21 and GPD1L expression in LUAD tissues analyzed by Pearson analysis. (f, g) The knockdown efficiency of miR-21 inhibitor on miR-21 expression in A549 (f) and H1299 (g) cells assessed by qRT-PCR, ^∗∗^*p* < 0.01*vs.* inhibitor. (h, i) The expression of GPD1L in A549 and H1299 cells after knockdown of miR-21 detected by qRT-PCR, ^∗∗^*p* < 0.01*vs.* inhibitor. (j, k) The effect of knockdown of miR-21 on the expression of GPD1L in A549 and H1299 cells detected by western blot. ^∗∗^*p* < 0.01*vs.* inhibitor.

**Figure 5:** miR-21 regulates the level of HIF-1*α* through GPD1L. (a, b) The expression of HIF-1*α* in A549 and H1299 treated by different concentrations of calycosin detected by qRT-PCR, ^∗∗^*p* < 0.01*vs*. control. (c, d) The expression of HIF-1*α* after knockdown of miR-21 or simultaneous knockdown of miR-21 and GPD1L (miR-21 inhibitor+si-GPD1L) in A549 and H1299 cells detected by qRT-PCR. (e, f) The protein expression of HIF-1*α* after knockdown of miR-21 or simultaneous knockdown of miR-21 and GPD1L (miR-21+si-GPD1L) in A549 and H1299 cells detected by western blot. (g) The correlation between GPD1L and HIF-1*α* expression in LUAD tissues analyzed by Pearson correlation analysis, ^∗∗^*p* < 0.01*vs.* inhibitor and ^##^*p* < 0.01*vs.* miR-21 inhibitor.

**Figure 6:** Calycosin regulates colony formation, invasion, migration, and EMT progression of LUAD cells through the circ0001946/miR-21/GPD1L/HIF-1*α* signaling axis. (a, b) The colony formation ability of A549 cells treated differently assessed by cell colony formation assay. (c, d) The invasion ability of A549 cells in each group detected by transwell. (e, f) The migration ability of A549 cells in each group determined by scratch assay. (g, h) The relative expression of EMT-related proteins (E-cadherin, N-cadherin, and Snail) of A549 cells in each group detected by western blot. (i, j) The mRNA expression of GPD1L (i) and HIF-1*α* (j) of A549 cells in each group determined by qRT-PCR. (k, l) The protein expression of HIF-1*α* of A549 cells in each group observed by western blot, ^∗∗^*p* < 0.01*vs.* control; ^##^*p* < 0.01 and ^#^*p* < 0.05*vs.* CA.

**Table 1:** Primers used for quantitative reverse transcription-polymerase chain reaction.

Gene name	Sequences (5′ to 3′)	Amplicon size
circ_0001946	F: TACCCAGTCTTCCATCAACTGG	121 bp
	R: ACACAGGTGCCATCGGAAAC	
miR-21	F: ACACTCCAGCTGGGTAGCTTATCAGACTGATG	67 bp
	R: TGGTGTCGTGGAGTCG	
GPD1L	F: CCGTGGTTGATGATGCAGACAC	110 bp
	R: CGCTTTGGTGTTGTCTCCACAG	
HIF-1*α*	F: TATGAGCCAGAAGAACTTTTAGGC	145 bp
	R: CACCTCTTTTGGCAAGCATCCTG	
GAPDH	F: GTCTCCTCTGACTTCAACAGCG	131 bp
	R: ACCACCCTGTTGCTGTAGCCAA	
U6	F: CTCGCTTCGGCAGCACA	75 bp
	R: AACGCTTCACGAATTTGCGT	

## Data Availability

The data used to support the findings of this study are available from the corresponding author upon request.
